# Evaluation of Football Teaching Quality Based on Big Data

**DOI:** 10.1155/2022/7174246

**Published:** 2022-06-28

**Authors:** Yue Long, Wei Zhai

**Affiliations:** Football College, Wuhan Sports University, Wuhan Hubei 430077, China

## Abstract

The arrival of the big data era has opened up new avenues for assessing the quality of physical education instruction. Using big data to explore these systems may help improve the quality of physical education itself, in addition to assisting schools in developing quality assessment systems for physical education. More and more schools are making football a compulsory part of their physical education and wellness curriculum. Therefore, this study used the methods of literature materials, expert interviews, questionnaires, and Delphi method to determine the evaluation indicators and index weight coefficients of football teaching and borrowed the application background of big data to initially explore the construction of a football teaching quality evaluation system. To this end, this paper completes the following tasks: (1) The current state of football teaching quality evaluation studies in the United States and internationally is summarized. (2) A football teaching quality evaluation system based on the background of big data is constructed. (3) Our experiments show that the assessment approach described in this study is scientifically and rationally distributed and can accurately represent all components of physical education. As a result, evaluating football instruction using big data is a possibility.

## 1. Introduction

Assessment of football instruction is a crucial step in football teaching. How and what evaluations are conducted have a direct bearing on the quality of high school football instruction, as well as the growth and development of PE instructors and their pupils. School football teachers are now evaluated mostly on their students' online feedback at the conclusion of each semester. A student's grade in physical education is based on their performance in class and on assessments given by the school itself. It is now time to get the physical education teacher's teaching score for this semester. As a result, the reform and growth of football instruction in schools in my nation is being held back by this paradigm [1]. Because of this, colleges and universities are increasingly focused on developing an assessment system for physical education instructors and students that allows for more active participation in the process of teaching feedback. There has been a dramatic rise of science and technology in our planet, the means of information circulation are becoming more and more diverse, and the amount of information exchange between people is growing rapidly. People in China and others can get real-time news, they can do online shopping through APPs such as Taobao and https://jd.com/, and they can inquire about all kinds of information they want through APPs such as Baidu and Zhihu. Therefore, under the background of the rapid popularization of mobile intelligent terminals, the vigorous development of mobile Internet, and the rise of the Internet of Things, big data is generated and developed. My country values big data innovation and incorporates it into its long-term growth objectives as a result of this strategy [2]. The introduction of big data applications has made it possible to automate the evaluation of physical education programs in schools. Physical education assessment may benefit from big data by providing a significant quantity of data support and, as a consequence, become more scientific and fair. Thanks to big data, physical education assessment can provide even more insight into the effectiveness of its methods. It is all about the technology here; it is all about the systems. The present physical education assessment system has been challenged by big data. A university that fulfills the needs of the big data age is reliable and operable and really supports the growth of students and physical education instructors and thus is required to be investigated. The assessment mechanism for physical education is essential. The purpose of this study is as follows:

1. To investigate and analyze the current situation of football teaching evaluation in some schools; the purpose is to solve the existing problems of the school football teaching evaluation system in our country and provide a small reference for the reform of the system
2. This research uses the Delphi method and AHP to determine the index and index weight coefficient of the football teaching evaluation system; its purpose is to provide a more reliable, scientific, and reasonable method for the determination of football teaching evaluation index and index weight coefficient
3. This study investigates the construction of a football teaching evaluation system using relevant big data knowledge in order to provide a new idea for the construction of a football teaching evaluation system, thereby promoting the implementation of sports teaching evaluation and providing relevant research. Through interdisciplinary research, this study applies the relevant knowledge of big data to football teaching evaluation, enriches the content of football teaching evaluation, and provides a certain reference for the study of football teaching evaluation

In addition, the study looks into using big data to create an assessment system for football instructors, as well as providing ideas and techniques for reforming the football teaching evaluation system in the age of big data. The value of this study lies in the timely feedback of the evaluation results of football teaching, so that physical education instructors are able to recognize the benefits and drawbacks of the teaching process and remedy them in time, thus enhancing the quality of education and instruction. The relevance and efficacy of football education are improved by helping schools adapt their objectives in a timely way. Students and instructors of physical education are enthused about sports evaluation, and schools are encouraged to use football evaluation, thereby promoting the process of reforming the physical education evaluation system [3]. This level is marked by equal attention to theory and practice, as well as the gradual adoption of behavioral features of physical education teachers' instruction as assessment indicators [4]. Third, in 1998, South Korea implemented the implementation evaluation method for primary school students, which comprehensively evaluated the changes and development of students' individual physical, mental, and athletic abilities [5–7].

The paragraph organization is as follows: Section 2 gives an overview of the related work.  Section 3 discusses the methods of the proposed concepts.  Section 4 discusses the experiments and results.  Section 5 concludes the article.

## 2. Related Work

There are many studies on physical education evaluation in China. As of February 2022, CNKI used “physical education evaluation” as the key word to retrieve more than 4,000 related literatures, including doctoral and master's theses, and journal literatures. It can be seen that the research on “physical education evaluation” has become a hot field of research today. This research has organized and analyzed the relevant materials collected. The assessment of domestic physical education instruction following my country's reform and opening up may be split into three stages: the first, the evaluation of instructors in this time; the second, the evaluation of students; and the third, the evaluation of programs. The school splits its assessment indicators into first- and second-level categories based on their degree of empirical support. Second, in the stage of regularization, the physical education evaluation in this period is more systematic, standardized, and open. Established in 1994, the Higher Education Research and Evaluation Association of the China Higher Education Society provides an organizational guarantee for teaching evaluation. This stage has the characteristics of paying equal attention to both theory and practice and gradually began to use the behavioral characteristics of physical education teachers' teaching as indicators for evaluation [4].

Now in 2001, a large number of academics have conducted a study on the assessment of physical education, and this evaluation has since spread throughout the nation. Teaching quality is an essential factor in the assessment of physical education teachers by colleges and universities [5]. As a result, several academics have turned their focus to the assessment of physical education (PE) teacher effectiveness. According to a review of the available literature, the majority of the international research on the assessment of physical education instruction has come from the United States, Japan, South Korea, Germany, and the United Kingdom. First, the physical education evaluation in the United States is mainly aimed at primary and secondary schools. Individual assessment should be used instead of a uniform evaluation standard in the evaluation of physical education. When it comes to evaluating students' performance and abilities in physical education in Japanese schools, pleasant sports are the norm, and this is reflected in the assessment of physical education, with thinking, judgment, knowledge, and understanding as the main content [6]. Third, in 1998, South Korea implemented the implementation evaluation method for primary school students, which comprehensively evaluated the changes and development of students' individual physical, mental, and athletic abilities [7]. Fourth, school sports in Germany attaches great importance to cultivating students' habit of self-exercise and strives to strengthen the communication and connection between school sports and social sports. Finally, the assessment of physical education in the United Kingdom emphasizes the need of developing students' initiative, awareness, and creativity [8]. Regarding the research status of big data in the field of sports, up to now, in the domestic research on big data, CNKI uses “big data” as the key word for retrieval, and the literature classification is set to “sports” to obtain more than 500 related documents. In 2012, my nation started to use big data-related expertise in sports research. Many sports researchers and academics in my nation have turned to big data applications since 2012, notably in the last three years. Many in the sports sector feel that by focusing on “big data,” the current age of big data will provide significant potential for the industry. The themes include “Big Data Era,” “Sports,” “Sports Industry,” “World Cup,” “Ball Games,” “Competitive Sports,” and “Sports Events.” In the fields of industry, competitive sports, and sports events, there are only 9 literatures on “physical education”; even fewer publications exist on the assessment of physical education.

According to some domestic researchers, contemporary civilization has made it easier to communicate knowledge. In a world of big data, it is possible to conduct a more scientific and unbiased assessment of college and university physical education programs since the quantity of data available has grown exponentially [9]. As a result, big data should be used to evaluate physical education in colleges and universities. To summarize, most research into the use of big data in sports in my country is theoretical, and there are few practical studies on the subject. Big data may be both an advantage and a hindrance when it comes to physical education assessment in my nation, where there is little research on football teacher evaluation. International research on the use of big data in sports is few and far between, but big data has been utilized in a variety of ways, and sporting events and sports are the most common. It has been shown that theoretical models of tactical decision-making in team sports benefit from contemporary machine learning and big data approaches. Reference [10] proposes a project aimed at introducing big data techniques into elite football research technical analysis. Volleyball teams may enhance their overall performance by using a computer-aided analysis tool (CAAT) to evaluate the underlying patterns that contribute to victories and defeats. Therefore, due to the scarcity of research in other countries on the use of big data for assessment in physical education, it is necessary for us to learn from other nations' experience with big data applications for other sports [11].

## 3. Method

In this section, we discuss the experimental method, construction of teaching quality evaluation system, weight distribution of teaching evaluation index system, and framework of evaluation system in the context of big data in depth.

### 3.1. Experimental Method

#### 3.1.1. Documentation Method

With the help of university libraries and Internet tools such as CNKI and Web of Science database, a large number of books, journals, and literature materials are consulted, and the consulted materials are organized to analyze physical education teaching evaluation, big data, and big data at home and abroad. According to the needs of the paper, we use “Physical Education Evaluation” and “Big Data” as the search keywords in CNKI (China National Knowledge Infrastructure) and “Big Data” in Web of Science. This paper focuses on 12 master's theses, 15 other documents, 3 foreign language documents, and 2 documents in the Web of Science database. *Architecting Big Data: Big Data Technology and Algorithm Analysis* and other books have provided a lot of precious inspiration and reference opinions, which provide reference and theoretical support for the research of this paper.

#### 3.1.2. Questionnaire Survey Method

Aiming at the current situation of teaching evaluation in a province, this paper selects physical education teachers and students from 5 schools to conduct a questionnaire survey on the relevant content of the implementation of sports evaluation. Six physical education teachers were selected from each school, and a total of 30 teachers were sent out for teacher questionnaires; each school selected 100 students, divided according to the ratio of boys and girls and grades, including 50 boys and 50 girls. By referring to the relevant literature, the first drafts of the questionnaires for physical education teachers and students were compiled. After listening to the suggestions of 100 experts and tutors, the contents of the questionnaires were revised, and the questionnaires were finally determined. Questionnaires were distributed to 30 physical education teachers and 500 students by way of face-to-face distribution. Its efficiency and recovery rate have reached 100%.

During this research, a questionnaire validity survey was done on 10 experts in the area of physical education in order to confirm its validity. Experts who thought the questionnaire design was reasonable accounted for 70% and 30% were basically reasonable. Therefore, the designed status questionnaire was basically recognized by experts, and its validity was high. In order to test the overall reliability of the questionnaire, the method of retest reliability was used. At an interval of 15 days, 5 copies of the teacher questionnaire and 10 copies of the student questionnaire were distributed again. The one-time coefficient of the current situation questionnaire for sports is 0.864, and the one-time coefficient of the current situation questionnaire for students is 0.811, both of which are >0.75, so the reliability of this questionnaire is high. In order to determine the indicators and weight coefficients of the school physical education teaching evaluation system, this paper conducted an indicator questionnaire survey and indicator weight consultation among 22 experts in the field of physical education. As a result of a thorough review of relevant literature and resources, as well as interviews with experts, accordingly, evaluation index and weight survey tables for the physical education teacher's teaching evaluation and the student's assessment of physical education were created. In both the teacher and student teaching evaluation index tables, there are three first-level indicators and fourteen second-level indicators for physical education introduction.

#### 3.1.3. Delphi and AHP

The Delphi method involves conducting two rounds of expert surveys among 22 experts in the field of physical education: the first round involves carefully analyzing and comparing the initially formulated indicators, assigning values based on the importance of each indicator by experts, performing the relevant consistency test, and finally making certain modifications to the indicators based on expert opinions. In the second round of expert survey, according to the assignment of the importance of each index by experts, the relevant consistency test was carried out. Using big data, the index method for evaluating college physical education teachers was eventually established [12].

To begin, a hierarchical structure model of college sports assessment indicators is created using big data, and then, the judgment matrix for each level is created. Check each level once more and then calculate the weight value of each indicator for each level. The weight value of the index is used to determine the degree of its influence on physical education assessment [13, 14].

### 3.2. Construction of Teaching Quality Evaluation System

#### 3.2.1. Characteristics and Principles of System Construction

With the rise of big data, the football teaching evaluation system may be reconstructed utilizing big data technology. Football teaching evaluation system qualities are outlined within the context of big data research and analysis: To begin, the appraisal is based on both personal experience and factual evidence. Second, the evaluation method changes from summative evaluation to accompanying evaluation. Third, the evaluation content is from singleness to diversity evaluation. Fourth, the evaluation methods have changed from manual evaluation to intelligent evaluation. The design of the football teaching assessment system should be founded on the theoretical foundation, beginning with all parts of the physical education process, and primarily satisfy the following guidelines:

1. The scientific and objective principles
2. The idea that everything should be included
3. The idea of bringing together commonalities and uniqueness in a harmonious way
4. The openness and timeliness of communication [15]

#### 3.2.2. Design of the System of Football Teaching Evaluation Indicators

Based on a study of physical education teaching evaluations in colleges and universities, a physical education teacher teaching evaluation index and a student physical education teaching evaluation index system might be constructed, as well as experts' recommendations and design principles for a big data-era evaluation system. This system is broken into three parts: the first- and second-level indices and descriptions of the indices in question. Physical education teachers' teaching evaluation index system contains 3 first-level indices, and students' teaching evaluation index system includes 3 first-level indices and 10 secondary indices. Using SPSS statistical software, we do parameter analysis on the computer to determine the relevance of each indicator in the assessment system, as assigned by 22 experts.

The response rate to the expert consultation form is measured by the expert excitement coefficient. The greater the response rate, the more excited the experts are about answering questions. The formula is as follows: *J* = *n*/*N*, where *N* is the total number of experts and *n* is the number of experts that participated. In this study, the recovery and effectiveness rates of the two rounds were 100% and 100% and 90.91% and 100%, respectively, which fulfilled the requirements of this research. The lower the coefficient of variation, the better the coordination of specialists [16]. If the standard deviation is greater than 0.25, it is considered that the degree of coordination is not high. The calculation formula is

(1) $$\begin{array}{c} V_{j}=\frac{S_{j}}{M_{j}}, \end{array}$$

(2) $$\begin{array}{c} M_{j}=\frac{1}{n}\overset{n}{\underset{j-1}{\sum }}X, \end{array}$$

(3) $$\begin{array}{c} S_{j}=\sqrt{\frac{1}{n-1}\overset{n}{\underset{i=1}{\sum }}{\left(X_{i}-M_{J}\right)}^{2}}, \end{array}$$

where *V*_*j*_ represents the coefficient of variation, *S*_*j*_ represents the standard deviation, and *M*_*j*_ represents the arithmetic mean, the smaller the coefficient of variation.

The Kendall harmony coefficient (KHC) *W* value can test whether the evaluation results of experts on the indicators are consistent. It is between 0 and 1, with higher values indicating more stability. When the *P* value is more than or equal to 0.05, the results are not consistent with Kendall's harmony coefficient; however, a *P* value of 0.05 indicates that the results are. The following is the formula for calculating the value:

(4) $$\begin{array}{c} W=\frac{S}{\left(1/12\right)\left[K^{2}\left(N^{3}-N\right)-K\sum_{i=1}^{K}T_{I}\right]}, \end{array}$$

(5) $$\begin{array}{c} S=\overset{n}{\underset{i=1}{\sum }}{\left(R_{i}-\bar{R_{i}}\right)}^{2}, \end{array}$$

(6) $$\begin{array}{c} T_{i}=\overset{M_{i}}{\underset{i=1}{\sum }}\left(N_{ij}^{3}-N_{ij}\right), \end{array}$$

(7) $$\begin{array}{c} X^{2}=K\left(N-1\right)W, \end{array}$$

where *N* represents the number of indicators evaluated, *K* represents the number of experts participating in the evaluation, *S* represents the sum of the grades of each evaluated indicator *R*_*i*_ and the average of all these sums $\bar{R_{i}}$ is the sum of squared deviations, and *T*_*i*_ represents the correction coefficient.

#### 3.2.3. Determination of the Evaluation Index System of Football Teaching

After two rounds of expert index questionnaire investigation and demonstration, data statistics, and analysis, we have finally figured out how to evaluate the physical education instructor (Table 1) and how to evaluate the student physical education teaching assessment system (Table 2).

### 3.3. Weight Distribution of Teaching Evaluation Index System

Using the Analytic Hierarchy Process (AHP), the weight coefficient of the evaluation index is calculated and determined. Using the analytic hierarchy approach, one may examine correlations between evaluation indicators, quantify the final findings, and then calculate each indicator's weight coefficient. The AHP technique is employed in order to establish the indicator weight, which assures that the indicator weight is reasonable and scientifically determined [17].

#### 3.3.1. Steps of the AHP Method

*(1) Build an Evaluation System*. Through two rounds of expert index questionnaire research, the obtained indices are analyzed.

*(2) Build a Hierarchy Model*. From the very top to the very bottom, the important indicators are categorized according to their many features and relative relevance.

*(3) Create a Judgment Matrix for the Results*. In order to create a judgment matrix, all evaluation indications are compared at the same level generally; the 1-9 scale method proposed by Saaty is used, such as the comparison of two indicators A and B.

*(4) Calculate the Weight Vector and Consistency Check*. The matrix's largest eigenvalue is max, and its formula is as follows: consistency ratio (CR) and consistency indicator (CI) are used in the calculation CR = CI/RI.

(8) $$\begin{array}{c} \lambda_{\max}=\frac{1}{n}\underset{i}{\sum }\frac{\left(\text{Aw}\right)i}{wi},\text{ CI}=\lambda_{\max}-\frac{n}{n-1}, \end{array}$$

where Aw is the product of the judgment matrix and the eigenvector and RI is the average random consistency index, which can be obtained through the difference table (see Table 3).

#### 3.3.2. An Evaluation Index's Weighted Coefficient May Be Calculated

The weight coefficient of the physical education teacher's teaching evaluation index is as follows: First, according to the Saaty 1-9 level judgment matrix standard degree table, the second round of the index weight consultation table, and 20 experts' scores, we establish the physical education teacher's teaching evaluation index system at all levels of judgment moments. Next, we enter the data of the judgment matrix of the first-level indicators in the Excel sheet and calculate the values of the in-row multiplication, the *n*-th power, the weight value  *W*, *λ*_max_, CI, CR, etc. The weights of the first-level indicators of the PE teacher's teaching evaluation index system are W1 = 0.12, W2 = 0.65, and W3 = 0.23. CR = 0.0036 < 0.1, so it indicates that the first-level index judgment matrix passes the one-time test. Finally, the weight coefficients of the remaining three rectangular matrices and the corresponding weight coefficients of the matrices established by the secondary indicators B1 to B14 are calculated in the Excel sheet according to the above method, and the weight table of the teaching evaluation index system for physical education teachers is obtained.

The weight coefficient of the student physical education evaluation index is as follows: using the above method, we calculate the weight table of the student physical education evaluation index system.

### 3.4. Framework of Evaluation System in the Context of Big Data

According to the subject, evaluation can be divided into two categories: one is self-evaluation and the other is evaluation of others [18]. Teaching and learning are two of the most important criteria in evaluating a teacher's ability to educate. Therefore, we should realize that different evaluation subjects have different roles at the process of developing an assessment system for physical education in colleges and universities and clarify the commonality and individuality among the subjects through evaluation indicators and indicator weights. In this study, we selected four evaluation subjects including physical education instructors, students, and other members of the school's physical education department. The specific framework is shown in Figure 1.

#### 3.4.1. Physical Education Evaluation Activities for Students

1. In this context, students' self-evaluation refers to students' self-awareness of their own learning process. Students who regularly do self-assessments have a better understanding of their own shortcomings and how to overcome them. As shown by the evaluation indicators, students perform an in-depth investigation of themselves as well as an overall assessment. The goal of this exercise is to help students better understand their learning preferences and methods, as well as their own strengths and shortcomings, to make the most of their own self-directed learning potential. Using your own teaching account, students may access a whiteboard for self-evaluation of their classroom experiences
2. Students are divided into equal groups for the purposes of group teaching assessment, and the group members use a one-to-one evaluation approach to assess each other's performance on the indicators. Additionally, kids will be more enthusiastic in sports learning as a result, as well as be able to share their own learning techniques with other students. It is thus possible to get additional information about how physical education is affecting the school's livestock by doing a group review. Students use the teaching evaluation account to rate their classmates in physical education classes. Teachers submit the information about the class ahead of time
3. Physical education teachers' evaluation activities: in the activities of physical education evaluation for students, physical education teachers are the subject of evaluation, whereas the focus is on the pupils themselves. Teachers' evaluations of pupils in physical education are the most authentic, clear, and convincing. PE instructors have the largest impact on students' physical education instruction. As a result, the assessment of physical education instructors is a critical component in assessing students' progress in physical education. In this study, physical education teachers can log in to the teacher system to evaluate physical education teaching for the students in their substitute classes

#### 3.4.2. Teaching Evaluation Activities for Physical Education Teachers

*(1) Physical Education Teachers' Self-Evaluation Activities*. The main approach of teaching quality evaluation is physical education instructors' self-evaluation, which refers to a physical education teacher's understanding of the quality of self-teaching. When PE teachers conduct self-evaluation, they can clearly recognize their own deficiencies in the process of physical education and improve themselves. Physical education teachers log in to the teacher system to conduct self-evaluation on their class situations.

*(2) Activity-Based Evaluations of Physical Education Instruction by Students*. Students and physical education teachers are in close touch, and student evaluations of physical education instructors are the most compelling. As a result, it is impossible to disregard the assessment actions of pupils. When evaluating student-taught sessions, it is critical to distinguish between physical education instructors and students. Students are the subject, and they take action against the teachers. Students can rate the physical education teacher's class using their teaching evaluation account.

*(3) Peer Evaluation of Teaching Activities*. Peer physical education instructors are the topic of the assessment process, while the assessed physical education teachers are the object of the evaluation procedure. There are no subjective evaluations in peer evaluations; thus, the individual physical education classroom survey is not taken into account by the peer instructors. Peer physical education teachers can conduct physical education teaching evaluation on physical education teachers by way of audition.

*(4) Teaching Evaluation Activities by the Personnel of the Competent Department of Physical Education*. First, the personnel of the competent department of physical education are familiar with the content and goals of physical education, and secondly, the personnel of the competent department of physical education can directly grasp the first-hand information of physical education teachers, so their evaluation is authoritative. Physical education department staff can evaluate physical education teachers' classes through random checks and auditions.

#### 3.4.3. Explore the Construction of Football Teaching Evaluation Process

Analysis of the present state of school teaching evaluation implementation shows that the assessment procedure for football is built on the use of big data. Teachers, administrators, and students are the primary beneficiaries of this tool. Collection, analysis, and interpretation of data make up the assessment process. In Figure 2, you can see the specifics of the output and result feedback in action.

## 4. Experiment and Analysis

In this chapter, we define the survey results and analysis of teacher evaluation indicators, survey results and analysis of student evaluation indicators, and indicator weight coefficient results in detail.

### 4.1. Survey Results and Analysis of Teacher Evaluation Indicators

Taking the evaluation results of the first- and second-level indicators of teachers by experts into the previous method for calculation, the following results were obtained: after two rounds of investigation, it was determined that the first-level indicators of football teachers' teaching evaluation included three items—the process of preparing to teach, the actual act of instructing, and the impact of that instruction. Preclass preparation, lesson plan composition, teaching etiquette, classroom routine, teaching attitude, teaching organization, teaching style, teaching material, and exercise load are secondary indicators used to evaluate football instructors, classroom atmosphere, sports skills, exercise awareness, and physical fitness; these are the 14 items of quality and theoretical basic knowledge. The parameter values of its primary and secondary indicators are shown in Figures 3 and 4.

Figure 3 shows that the parameters of the first-level indicators of teachers' teaching evaluation all exceed 4. Among them, the parameters of the teaching process and teaching effect even exceed 4.5, which show that experts have a high degree of recognition of these two items. Secondly, the Kendall harmony coefficient was 0.42, with a *P* value of 0.05 suggesting a substantial and well-coordinated set of expert evaluations. Teaching preparation, teaching method, and teaching impact are the three primary measures used to evaluate the effectiveness of football instructors in the classroom.  Figure 4 shows that the parameters of the secondary indicators of teacher teaching evaluation also exceed 4, indicating that 14 secondary indicators have been recognized by experts. Secondly, the Kendall harmony coefficient rose to 0.35, which was greatly improved compared with the first round, indicating that the expert opinions were more coordinated. The chi-square value was 92.19, and the significance test *P* was much less than 0.05, indicating that the expert evaluation results were consistent. Finally, the secondary indicators of teacher teaching evaluation are these 14 items, and the consistency test statistical table of the primary and secondary indicators is shown in Table 4.

### 4.2. Survey Results and Analysis of Student Evaluation Indicators

After two rounds of investigation, it was determined that the first-level indicators of students' football teaching evaluation were learning preparation, learning process, and learning effect. Preclass preparation, learning etiquette, classroom routine, learning attitude, emotional cooperation spirit, classroom atmosphere, sports skills, training awareness, physical quality, and basic knowledge of sports theory are the secondary indicators used to determine students' physical education teaching evaluation. The comparison of its primary and secondary index parameters is shown in Figures 5 and 6.

Figure 5 shows that after two rounds of investigation, the parameters have obvious changes. The average of the three indicators of learning preparation, learning process, and learning effect increased, and the coefficient of variation decreased. Among them, the index of learning preparation increased “learning etiquette,” the mean increased to 4.05, and the coefficient of variation decreased to 0.19. The mean of the effect index increased to 4.55, and the coefficient of variation decreased to 0.11. Secondly, according to the Kendall harmony coefficient, the assessment findings of experts were coordinated and consistent. The Kendall harmony coefficient achieved 0.45, *P*0.05. Finally, we determine the first-level indicators of students' PE teaching evaluation as learning preparation, learning process, and learning effect. This is shown by Figure 6. The averages of all indicators evaluated by students are all over 4, and the coefficients of variation are all less than 0.25, indicating that after these two rounds of expert indicator questionnaire surveys, experts have detected all ten secondary indications. First of all, the Kendall harmony coefficient shows that the expert survey findings are well coordinated, with a value of 0.44; the chi-square value is 81.63; and the significance test *P* is less than 0.05, indicating that the expert survey results are significant. Finally, we determine the secondary indicators of students' PE teaching evaluation as these 10 items. The consistency test of the primary and secondary indicators of student physical education teaching evaluation is shown in Table 5.

### 4.3. Indicator Weight Coefficient Results

The weights of various indicators of teachers and students in football teaching are calculated by the AHP method mentioned above, as shown in Tables 6 and 7.

## 5. Conclusion

In the current state of school physical education evaluation, there are numerous challenges that divert from the original intent of the discipline, including a single subject and model, unscientific techniques, a lack of originality in standards, an inadequate assurance system, and an unsatisfactory feedback mechanism; all contribute to the lack of individuality in standards. As a result, it is inextricably related to my country's long-established, centralized, and consistent educational administration structure. The study's index weight coefficient distribution is more scientific and sensible because big data was used to construct evaluation indicators that could reflect practically every aspect of football instruction. As a result, big data can be utilized to assess physical education. The bulk of persons being evaluated for their work in the field of physical education in the context of big data applications is physical education instructors, students, peers, and employees in physical education departments. Data collection, data analysis, result output, and feedback are all components of a school physical education teaching evaluation system. In order to get reliable findings, data collection must be thorough, data analysis must be scientific, and feedback must be prompt and accurate. The assessment of physical education is incomplete without each connection.

## Figures and Tables

**Figure 1:** Framework of football teaching evaluation system.

**Figure 2:** Football teaching evaluation process.

**Figure 3:** Comparison of the first-level index parameters of teacher evaluation (*N* = 20).

**Figure 4:** Second-level index parameters of teacher teaching evaluation (*N* = 20).

**Figure 5:** Comparison of primary indicators of student evaluation.

**Figure 6:** Comparison of secondary indicators of student evaluation.

**Table 1:** Physical education teacher teaching evaluation index system.

First-level indicator	Secondary indicators
Teaching preparation A1	Preparation before class B1
	Lesson plan writing B2
	Teaching etiquette B3
	Classroom routine B4
	Teaching attitude B5
Teaching process A2	Teaching organization B6
	Teaching methods B7
	Teaching content B8
	Exercise load B9
	Classroom atmosphere B10
Teaching effect A3	Exercise awareness to develop B11
	Soccer skills B12
	Physical fitness B13
	Basic knowledge of sports theory B14

**Table 2:** Student football teaching evaluation index system.

First-level indicator	Secondary indicators
Learn to prepare C1	Preparation before class D1
	Teaching etiquette D2
Learning process C2	Classroom routine D3
	Learning attitude D4
	Cooperative spirit D5
	Classroom atmosphere D6
Learning effect C3	Exercise awareness to develop D7
	Soccer skills D8
	Physical fitness D9
	Basic knowledge of sports theory D10

**Table 3:** RI value table.

Order	1	2	3	4	5	6	7	8	9	10
RI	0.00	0.00	0.59	0.91	1.13	1.22	1.33	1.53	1.46	1.50

**Table 4:** Consistency test of primary and secondary indicators.

Index	KHC	Chi-square value	*P* value
First-level indicator	0.43	17.84	0.0002 < 0.05
Secondary indicators	0.37	92.19	<0.05

**Table 5:** Consistency test of primary and secondary indicators.

Index	KHC	Chi-square value	*P* value
First-level indicator	0.45	18.14	0.0002 < 0.05
Secondary indicators	0.44	81.63	<0.05

**Table 6:** The weight of teachers' primary and secondary indicators.

First-level indicator	Index weight	Secondary indicators	Index weight
A1	0.13	B1	0.16
		B2	0.74
		B3	0.11
		B4	0.01
		B5	0.12
A2	0.67	B6	0.25
		B7	0.23
		B8	0.24
		B9	0.07
		B10	0.04
A3	0.20	B11	0.06
		B12	0.32
		B13	0.57
		B14	0.05

**Table 7:** Weights of primary and secondary indicators of students.

First-level indicator	Index weight	Secondary indicators	Index weight
C1	0.07	D1	0.76
		D2	0.24
C2	0.65	D3	0.12
		D4	0.20
		D5	0.60
		D6	0.08
C3	0.28	D7	0.13
		D8	0.30
		D9	0.46
		D10	0.11

## Data Availability

The datasets used during the current study are available from the corresponding author on reasonable request.
